The article "Roles of Epigenetic Modifications in the Differentiation and Function of Pancreatic β-Cells" was retracted in 2022. Reasons: plagiarism; overlap with other authors' work.

# Roles of Epigenetic Modifications in the Differentiation and Function of Pancreatic β-Cells

**DOI:** 10.3389/fcell.2020.00748

**Published:** 2020-08-28

**Authors:** Fei Xu, Jing Liu, Lixin Na, Linjun Chen

**Affiliations:** ^1^Department of Microbiology and Immunology, Shanghai University of Medicine & Health Sciences, Shanghai, China; ^2^Collaborative Innovation Center of Shanghai University of Medicine & Health Sciences, Shanghai, China; ^3^Department of Inspection and Quarantine, Shanghai University of Medicine & Health Sciences, Shanghai, China

**Keywords:** epigenetics, pancreatic β cells, histone modification, DNA methylation, non-coding RNA

## Abstract

Diabetes, a metabolic disease with multiple causes characterized by high blood sugar, has become a public health problem. Hyperglycaemia is caused by deficiencies in insulin secretion, impairment of insulin function, or both. The insulin secreted by pancreatic β cells is the only hormone in the body that lowers blood glucose levels and plays vital roles in maintaining glucose homeostasis. Therefore, investigation of the molecular mechanisms of pancreatic β cell differentiation and function is necessary to elucidate the processes involved in the onset of diabetes. Although numerous studies have shown that transcriptional regulation is essential for the differentiation and function of pancreatic β cells, increasing evidence indicates that epigenetic mechanisms participate in controlling the fate and regulation of these cells. Epigenetics involves heritable alterations in gene expression caused by DNA methylation, histone modification and non-coding RNA activity that does not result in DNA nucleotide sequence alterations. Recent research has revealed that a variety of epigenetic modifications play an important role in the development of diabetes. Here, we review the mechanisms by which epigenetic regulation affects β cell differentiation and function.

## Introduction

The global incidence of diabetes has risen sharply with societal progress and improvements in living standards, and the disease is showing a trend toward affecting younger individuals. At present, ~1/10th of the world's medical expenses are used for the treatment of diabetes and its complications, imposing heavy economic burdens on patients' families and on society as a whole (Hassan et al., 2017). Diabetes and its complications are common and challenging global problems in the twenty-first century. Diabetes, which is a chronic metabolic disease characterized by elevated blood sugar, is caused by the interaction of multiple factors, including genetic, environmental, social, and psychological factors, and among others (Kolb and Martin, 2017). Persistent hyperglycaemia causes chronic damage to various organs, including the eyes, kidneys, heart, blood vessels, and nerves, which can eventually lead to patient death due to organ failure (Zimmet et al., 2016). According to the pathogenesis, diabetes is mainly divided into two types: Type 1 diabetes (T1D) is caused by an autoimmune attack targeting the insulinproducing pancreatic b-cells, while type 2 diabetes (T2D) is associated with aging, early development of insulin resistance, and a deteriorating β cell function. T2DM is a complex disease resulting from the interaction of genetic, epigenetic, environmental, and lifestyle factors. About 90% of diabetic cases worldwide are accounted to be T2D and predominantly targets adults. Furthermore, T2DM can be complicated with chronic conditions, such as hypertension, coronary heart disease, stroke, macrovascular and microvascular complications, which has greatly challenged the global medical and health system; thus, the prevention and treatment of diabetes and its complications have become popular research topics worldwide (Ueda et al., 2019).

The article "Roles of Epigenetic Modifications in the Differentiation and Function of Pancreatic β-Cells" was retracted in 2022. Reasons: plagiarism; overlap with other authors' work.

Epigenetics was originally proposed by Waddington in 1942, and its definition was finalized at the 2008 Cold Spring Harbor Conference as “a stable heritable phenotype caused by chromosomal changes without changing the DNA sequence” (Berger et al., 2009; Waddington, 2012). Researches have revealed that the mechanisms of these changes mainly comprise DNA methylation, histone modification and noncoding RNA (ncRNA) activity (Ling and Ronn, 2019). Epigenetic regulation exists throughout the lifetime of an organism and participates in many life activities. Any abnormality in the epigenetic regulatory mechanism will affect chromatin structure and gene expression, leading to the occurrence of a variety of diseases (Nilsson et al., 2018; Li S. et al., 2019; Perez and Lehner, 2019). Epigenetic changes are important regulatory mechanisms of islet β cell function and play irreplaceable roles in the normal physiological function of pancreatic β cells and insulin-secreting cells and apoptosis (Courty et al., 2019; Gong and Jiang, 2020; Makkar et al., 2020). There is no doubt that epigenetics research already becomes the focus of the study of pancreatic β cells in recent years. Epigenetic modifications are closely related to other biological processes in the physiological function of pancreatic β cells. If the epigenetic changes are moderately induced or controlled by drug intervention, it is expected to become a new point to prevent the occurrence and development of diabetes.

## Effects of Dna Methylation on β Cell Differentiation and Function

DNA methylation modification is by far the most thoroughly studied epigenetic modification (Shafabakhsh et al., 2019). DNA methylation modification is mainly controlled by DNA methyltransferase (DNMT) family proteins (Table 1) (Sahin et al., 2010). S-adenosylmethionine is used as the methyl donor to methylate the cytosine on CpG islands. Normally, the CpG island of a gene is in an unmethylated state. Methylation of the cytosines in the CpG island can inhibit the expression of this gene (Figure 1). Increasing evidence shows that the regulation of methylation level is related to diet, physiological activities and glucose level, indicating that methylation is a dynamic process (Wicklow and Sellers, 2015). There is evidence that both the density and methylation level of tissue-specific promoter CpG islands play important roles in the regulation of gene expression (Bansal and Pinney, 2017; Ponnaluri et al., 2017; Zhou et al., 2018).

The article "Roles of Epigenetic Modifications in the Differentiation and Function of Pancreatic β-Cells" was retracted in 2022. Reasons: plagiarism; overlap with other authors' work.

**Table 1:** Members and functions of DNA methylated transferases.

**Name**	**Location**	**Functions**
DNMT1	19p13.2	The main enzyme to maintain methylation which ensures the normal replication of DNA methylation mode; and also necessary for de methylation of non CpG sites (Tajima et al., 2016)
DNMT2	10p15.1	The methyltransferase of aspartic tRNA, which can methylate 38°C of aspartic tRNA (Goll et al., 2006)
DNMT3A	2p23.3	The main *de novo* DNA methyltransferase which establishes DNA methylation patterns in gametes and early embryos (Chedin, 2011; de Mendoza et al., 2018)
DNMT3B	20q11.2	The main *de novo* DNA methyltransferase which establishes DNA methylation patterns in gametes and early embryos (Chedin, 2011)
DNMT3L	21q22.3	Has no methyltransferase activity by itself, interacts with the DNMT3A and DNMT3B catalytic regions to enhance the activity of DNMT3A and DNMT3B, thus facilitating *de novo* methylation (Chedin, 2011)

*DNMT1, DNA methyltransferase 1; DNMT2, DNA methyltransferase 2; DNMT3A, DNA methyltransferases 3A; DNMT3B, DNA methyltransferases 3B; DNMT3L, DNA methyltransferases 3L*.

**Figure 1:** Molecular mechanism of DNA methylation (Bansal and Pinney, 2017; Ponnaluri et al., 2017; Zhou et al., 2018; Shafabakhsh et al., 2019). DNA methylation modification is mainly controlled by DNMT proteins. S-adenosylmethionine is used as the methyl donor to methylate the cytosine on CpG islands. Normally, the CpG island of a gene is in an unmethylated state. Methylation of the cytosines in the CpG island can inhibit the expression of this gene.

### DNA Methylation in Diabetic Patients

Both the environment and diet can lead to apparent changes in the modification of certain imprinted genes and transposable elements in the genome, which in turn affect the development of the disease (Jirtle and Skinner, 2007). Research has shown that glucose metabolism disorders in T2DM patients are related to the hypomethylation of DNA in peripheral blood leukocytes (Toperoff et al., 2015). Another example is in adults exposed to famine during the Dutch Hunger Winter in the late period of World War II. The offspring of these individuals presented a low-birth weight, as well as an increase in the incidence of obesity, T2DM and dyslipidemia (Barres and Zierath, 2016). The DNA methylation level of genes related to cardiovascular disease in peripheral blood leukocytes of diabetic patients was significantly higher than that of normal people, and the DNA methylation level in saliva of diabetic nephropathy patients was significantly higher than that of ordinary people (Babu et al., 2015; Ronn and Ling, 2015). In addition, studies have shown that the long-term exposure of insulin and glucose will seriously change the DNA methylation status of skeletal muscle, indicating that DNA methylation is a rapid adaptation epigenetic marker (Mudry et al., 2017).

The article "Roles of Epigenetic Modifications in the Differentiation and Function of Pancreatic β-Cells" was retracted in 2022. Reasons: plagiarism; overlap with other authors' work.

The methylation of the CpG island in the insulin promoter region may play a crucial role in the maturation and tissue-specific expression of insulin genes in pancreatic β cells. Research scholars at Malmö University Hospital in Sweden found that in the islets of T2DM patients and those of non-T2DM donors, insulin promoter DNA methylation in human islets was negatively correlated with insulin gene expression and positively correlated with HbA1c (Yang et al., 2011). Relatedly, insulin methylation levels increased and expression decreased in T2DM patients (Yang et al., 2011). Dayeh et al. performed DNA methylation chip array analysis on islets donated by 15 T2DM patients and 34 normal controls and found that 853 genes and 1,649 CpG sites were differentially methylated in the islets of diabetic patients (Dayeh et al., 2014). *In vitro* experiments confirmed that methylation of the CDKN1A and PDE7B promoter genes inhibited their transcriptional activity and led to a decrease in the exocytosis function of pancreatic β cells and reduced insulin secretion (Dayeh et al., 2014). These epigenetic changes provide further insight into the pathogenesis of diabetes.

### DNA Methylation in β Cell Differentiation and Function

The role of DNA methylation in early pancreatic development is unclear, and Anderson et al. found in a model of induced pancreatic β cell ablation that DNA methylation in pancreatic progenitor cells plays an important role in the differentiation of pancreatic progenitor cells (Anderson et al., 2009). The specific knockout of DNMT1 in mouse pancreatic progenitor cells showed pancreatic progenitor cell apoptosis and pancreatic hypoplasia (Georgia et al., 2013). In mature β cells, defects in DNMT1 or DNMT3 can cause β cells to lose their “identity” and be reprogrammed into alpha cells, indicating that inhibition of alpha cell programming is necessary to maintain the “identity” of β cells (Dhawan et al., 2011). Currently, research has found that the occurrence of this reprogramming is related to the methylation of the Aristaless-related homeobox (Arx) promoter, causing abnormal Arx expression in β cells (Dhawan et al., 2011). In β cells, the inhibition of this methylation mediator ArxTat occurs through the interaction of NK2 homeobox 2 (Nkx2.2) with an inhibitory complex containing Grg3 (also known as Tle3), HDAC1 and Dnmt3A (Papizan et al., 2011). Therefore, in current cell replacement therapy research, endogenous alpha cells are considered to be important for β cell reprogramming. Recent studies have also shown that inhibiting DNA methylation in pancreatic progenitor cells promotes alpha cell production (Liu et al., 2019). In addition, the hypermethylation of CpG islands can reduce the expression of HNF4α gene and affect the differentiation of pancreatic β cells (Gilbert and Liu, 2012).

The article "Roles of Epigenetic Modifications in the Differentiation and Function of Pancreatic β-Cells" was retracted in 2022. Reasons: plagiarism; overlap with other authors' work.

PDX1 mutations can cause special types of diabetes, showing that PDX1 silencing can promote pancreatic β cell damage leading to diabetes (Pedica et al., 2014). The DNA methylation of 10 CpG sites in the PDX1 promoter and enhancer regions of pancreatic islets in T2DM patients was increased compared with the control group. Pancreatic β cells exposed to hyperglycaemia showed increased DNA methylation and decreased expression of PDX1 in the islets. Overall, the epigenetic modification of PDX1 may play a role in the development of T2DM.

Peroxisome proliferator-activated receptor γ coactivation 1α (PPARGG1α) is a transcriptional coactivator with high levels of expression in the human liver, kidneys, pancreas and skeletal muscles. DNA methylation of the PPARGG1α promoter may be an important cause of diabetic cardiopathy (Lacquemant et al., 2000; Waldman et al., 2018). Ling et al. reported that the DNA methylation of the PPARGG1α promoter in the islets of T2DM patients was accompanied by decreased mRNA expression, suggesting that epigenetics can regulate the expression of the PPARGG1α gene and subsequently affect insulin secretion (Ling et al., 2008).

TCF7L2 is a T2DM susceptibility gene that can promote the proliferation and survival of pancreatic β cells, and regulate the function of glucagon-like peptide (GLP-1) synthesis by intestinal L cells. Hu et al. performed high-throughput detection on pancreatic islet cells cultured in high fat and high glucose and found that chronic glycolipid toxicity can induce abnormal DNA methylation of the TCF7L2 gene, which may be one of the mechanisms of glycolipid toxicity leading to the deterioration of diabetic islet cells (Hu et al., 2014).

The article "Roles of Epigenetic Modifications in the Differentiation and Function of Pancreatic β-Cells" was retracted in 2022. Reasons: plagiarism; overlap with other authors' work.

In addition, DNA methylation is considered to be an important intergenerational genetic mechanism (Sarkies, 2020). DNA methylation markers in paternal and maternal genomes undergo reprogramming during mammalian fertilization and embryonic development; however, some imprinted genes escape the demethylation process during this time and thus change the representative type, resulting in intergenerational inheritance. In 2015, a study of perinatal female rat (F0) exposured to bisphenol A showed that the methylation of the imprinted gene insulin-like growth factor 2 (Igf2) of the F2 generation can be changed and cause intergenerational inheritance to impaire insulin secretion and glucose intolerance of the offspring (Mao et al., 2015). Su Rina et al. established a rat model of moderate intrauterine hyperglycemia induced by streptozotocin to detect glucose and lipid metabolism of first-generation (F1) and second-generation (F2) offspring. The results showed that F1 and F2 offspring which were exposed to intrauterine hyperglycemia had impaired insulin secretion from the islets, and both F1 and F2 offspring showed similar hypomethylation level at the−1952 site of the tumor necrosis factor (Tnf) gene (Su et al., 2016). These results confirmed that DNA methylation occurs in offspring exposed to intrauterine hyperglycemia and that the DNA methylation is intergenerational and inherited.

Ten eleven translocation (TET) enzymes and thymine DNA glycosylase (TDG) are implicated in active DNA demethylation (Ito et al., 2010). The three TET family enzymes oxidize 5-methylcytosine (5mC) in DNA to 5-hydroxymethylcytosine (5hmC), and subsequently to 5-formylcytosine (5fC) and 5-carboxylcytosine (5caC) (Ito et al., 2010; He et al., 2011). TDG, a base excision repair glycosylase, replaces 5fC and 5caC with an unmodified cytosine via DNA repair (He et al., 2011). Although recent data suggest a role of TET and 5hmC in embryonic stem cells and primordial germ cells, evidence for enzymatic demethylation by TET enzymes during differentiation of cells of later stages, such as the postnatal and adult stem cells of various organs including pancreas, remains very limited (Auclair and Weber, 2012; Tan and Shi, 2012). Interestingly, TET2 and TET3 are highly expressed in the murine adult pancreas, yet the pancreas has lower genomic 5hmC levels than other adult tissues derived from endoderm, including liver and lung (Ito et al., 2010, 2011), suggesting dynamic DNA demethylation during pancreas development. Xianghui Fu et al. found that TETs and TDG are direct targets of miR-26a and the expression of TETs and miR-26a change in opposite directions during *in vivo* and *in vitro* pancreatic cell differentiation (Fu et al., 2013). Another study showed that IFN-α exposure causes DNA demethylation by upregulation of the exoribonuclease PNPase old-35 (PNPT1), which mediates degradation of miR-26a leading to overexpression of methylcytosine dioxygenase TET2 and increased 5-hydroxymethylcytosine levels in human islets and β cells. These results provide a mechanistic framework to explain how inflammatory triggers such as viral infections can modify the β cell epigenome and modulate the interactions between the immune system and β cells (Stefan-Lifshitz et al., 2019). Therefore, the role of dynamic DNA demethylation during pancreas development deserves further study.

The article "Roles of Epigenetic Modifications in the Differentiation and Function of Pancreatic β-Cells" was retracted in 2022. Reasons: plagiarism; overlap with other authors' work.

## The Role of Histone Modification in β Cell Differentiation and Function

The core histones in the chromatin structure are subject to a series of covalent modifications with different chemical groups (including acetylation and methylation) that lead to the formation of a modified cascade called a histone code. The histone code can be recognized by a series of protein complexes, is translated into a specific chromatin state, and has a very important gene transcription regulatory function (Sims and Reinberg, 2008). The ease of access to the transcription factor binding site on chromatin is determined by the position and encapsulation of histones, and the degree of nucleosome compression is determined by the activity of a series of enzymes that are responsible for various histone-specific covalent modifications (such as acetylation, methylation, and phosphorylation) (Berger, 2007). The most studied types of histone modifications are acetylation and methylation of specific amino acid residues of histones H3 and H4 (Figure 2). Related research shows that during the differentiation and development of β cells, histone modification plays an important regulatory role and can recruit protein complexes to participate in the regulation of the expression of related genes in β cells (Ahmed et al., 2017; Balaji et al., 2018; Makkar et al., 2020).

**Figure 2:** Molecular mechanism of histone modification (Ahmed et al., 2017; Balaji et al., 2018; Makkar et al., 2020). **(A)** The histone acetylation process consists of HATs and HDACs. HATs can catalyse histone acetylation, resulting in the relaxation of chromatin structure, and makes it easy to recruit transcription factors to combine with them and promote the transcriptional expression of genes. On the contrary, HDACs deacetylate histones to lead to chromatin compression and inhibit gene transcription. HATs and HDACs jointly participate in the dynamic equilibrium processes of histone acetylation to precisely regulate gene transcription, such as for histone H3 at positions 9, 14, 18, and 23. Once the dynamic equilibrium state of acetylation and deacetylation of histones is broken, it may cause disease. **(B)** Histone methylation often occurs at the lysine or arginine residues of histone H3 and H4. Histone methylation is more stable and persistent than histone acetylation. Histone methylation of different forms and at different amino acid sites can lead to activation or inhibition of gene transcription. The forms of histone methylation include monomethylation, dimethylation, and trimethylation. Histone lysine methylation is relatively stable and often occurs at positions H3K4, H3K9, H3K27, H3K36, and H3K79.

The article "Roles of Epigenetic Modifications in the Differentiation and Function of Pancreatic β-Cells" was retracted in 2022. Reasons: plagiarism; overlap with other authors' work.

### Histone Methylation

Histone methylation often occurs at the lysine or arginine residues of histone H3 and H4. Such methylation is cocatalysed by histone methyltransferases (HMTs) and histone demethylase 1 (lysine demethylase 1, LSD1), indicating that the histone methylation process is reversible (Jenuwein, 2006). Histone methylation is more stable and persistent than histone acetylation. Histone methylation of different forms and at different amino acid sites can lead to activation or inhibition of gene transcription (Marmorstein and Trievel, 2009). The forms of histone methylation include monomethylation, dimethylation, and trimethylation. Histone lysine methylation is relatively stable and often occurs at positions H3K4, HK9, H4K20, H4K27, H3K36, and H3K79 (Table 2).

**Table 2:** Histone-lysine methyltransferase in the differentiation and function of pancreatic β cells.

**Genes**	**Action sites**	**Targets**	**Functions**
EHMT2 or G9a	H3K9me3, H3K27	HMGA1	Gene silencing (Cao et al., 2019)
SETDB1	H3K9me3	PPARγ, CEBPα	Gene silencing (Okamura et al., 2010)
SET7/9	H3K4	HIF-1α,	Gene silencing (Baek and Kim, 2016)
		p21, PDX1, BETA2	Gene activation (Maganti et al., 2015)
SET8	H4K20	/	Block ROS accumulation, attenuat vascular inflammation, and restore nitric oxide production (Yao et al., 2014)
PRC2	H3K27	Insulin gene	Inhibit the expression of insulin (Pethe et al., 2014)
		RAD21	Increased MafA expression (Deering et al., 2009)
		PDX1	Inhibit the differentiation of β cells (Chang et al., 2016)
		LncRNA ANRIL	Increased VEGF expression (Thomas et al., 2017)
		miR-200b	Increased VEGF expression (Ruiz et al., 2015)
SUV39H1	H3K9	p53	Gene silencing (He et al., 2012)
KMT2D/MLL2	H3K4	/	Regulate glucose homeostasis (Scoville et al., 2015)
KMT2C/MLL3			
KMT2B/MLL4			
NSD2	H3K36	PDX1	Promote the differentiation of β cells (Poulin et al., 2016)
EZH2	H3K27me3	INK4a/ARF	Gene silencing (Chen et al., 2009)

*HMGA1, high mobility group at-hook 1; BDNF, brain derived neuro trophic factor; PPARγ, peroxisome-proliferator activated receptor γ; CEBPα, CCAAT-enhancer binding protein α; HIF-1α, hypoxia inducible factor-1α; PDX1, pancreatic and duodenal homeobox 1; BETA2, beta cell E-box transcription factor 2; SUV39H1, suppressor of variegation 3-9 homolog 1; KMT2D, lysine methyltransferase 2D; KMT2B, lysine methyltransferase 2B; KMT2C, lysine methyltransferase 2C; NSD2, nuclear receptor binding SET domain protein 2; EZH2, enhancer of zestehomolog 2; INK4a/ARF, inhibitor of CDK4/ alternative reading frame*.

The article "Roles of Epigenetic Modifications in the Differentiation and Function of Pancreatic β-Cells" was retracted in 2022. Reasons: plagiarism; overlap with other authors' work.

### Histone Acetylation

The histone acetylation process consists of histone acetyltransferases (HATs) and histone deacetylases (HDACs) (Ahmed et al., 2017). It is known that HATs can catalyse histone acetylation, resulting in the relaxation of chromatin structure, and makes it easy to recruit transcription factors to combine with them and promote the transcriptional expression of genes. On the contrary, HDACs deacetylate histones to lead to chromatin compression and inhibit gene transcription. HATs and HDACs jointly participate in the dynamic equilibrium processes of histone acetylation to precisely regulate gene transcription, such as for histone H3 at positions 9, 14, 18, and 23 (Gilbert and Liu, 2012). Once the dynamic equilibrium state of acetylation and deacetylation of histones is broken, it may cause disease. It was previously shown that the level of H3K9 acetylation in the promoter region of insulin receptor substrate 2 (IRS2) was positively correlated with the expression level of IRS2 in pancreatic β cells (Kawada et al., 2017). High expression of HDAC7 impairs the secretory ability of rat islet cells, and the expression level of islet HDAC7 in T2DM patients is significantly increased compared with healthy group (Daneshpajooh et al., 2017).

### Histone Deacetylase Inhibitors (HDACis) and Pancreatic β Cells

HDACis can improve the function of pancreatic β cells, promote insulin synthesis and release, reduce inflammatory response-induced damage to pancreatic β cells, regulate the influence of the systemic immune response on T1DM and T2DM, and ameliorate the complications of diabetes (Sharma and Taliyan, 2016a). Short-chain fatty acids (such as butyric acid) that act as HDACis are intestinal fermentation products that exist in natural foods and may have broad application prospects in the treatment of GDM.

HDACis can be divided into 6 categories, according to their chemical structure (Table 3): ➀ short-chain fatty acids, such as sodium valproate (VPA) and sodium butyrate (NaB);➁ hydroxamic acids, such as trichostatin A (TSA) and suberoylanilide hydroxamic acid (SAHA); ➂ cyclic tetrapeptides, such as trapoxin A, (TPX); ➃ benzamides, such as entinostat (MS-275); ➄ epoxy ketones, such as trapoxin B; and ➅ hybrid molecules, such as peptide hydroxamic acids (cyclic hydroxamic acid-containing peptide 31, CHAP31) (Christensen et al., 2011; Sharma and Taliyan, 2016a). Mosley et al. verified the effect of glucose concentration on the acetylation of the insulin gene promoter in the islet β cell line MIN6. Their study revealed that the histone acetylation level of the glucose promoter was significantly greater when the glucose concentration was 30 mmol/L than when it was 3 mmol/L. After treatment with the HDACi TSA, the degree of H3 and H4 acetylation on the insulin gene promoter in the 3 mmol/L glucose group was similar to that in the 30 mmol/L glucose group, and the mRNA expression of insulin in the cells cultured with glucose was similar. These results show that TSA and NaB can promote insulin promoter histone acetylation to accelerate insulin transcription (Mosley et al., 2004). In addition, studies have found that IL-1, TNF-α and other inflammatory cytokines are closely related to islet cell damage and can affect the expression of multiple genes in pancreatic β cells, including cell apoptosis, cell cycle regulation, cell differentiation and metabolism (Ortis et al., 2010). After HDACi intervention, IL-1β- or TNF-α-induced apoptosis of cultured β cells *in vitro* is inhibited, which protects pancreatic β cells from cytokine toxicity. HDACis bind to oligonucleotides to form complexes that reduce the transcription of NF-κB-dependent genes, such as inducible nitric oxide synthase (iNOS) and NF-κB inhibitor genes (Larsen et al., 2007; Lundh et al., 2010). In animal models of diabetes, the inflammatory response can inhibit the survival of pancreatic β cells, and many HDACis (e.g., TSA and SAHA) can reduce cytokine-induced inhibition of insulin secretion. Inhibiting the inflammatory response is considered a key step in patients undergoing pancreatic β cell transplantation for diabetes (Lundh et al., 2010).

The article "Roles of Epigenetic Modifications in the Differentiation and Function of Pancreatic β-Cells" was retracted in 2022. Reasons: plagiarism; overlap with other authors' work.

**Table 3:** Effects of HDACis in preclinical animal models of insulin resistance.

**HDAC inhibitor**	**Dosage regimen**	**Animal model**	**Potential benefit**
NaB	5% w/w for 16 weeks	HFD-fed mice	Increased insulin sensitivity; Increased energy expenditure (Gao et al., 2009)
	500 mg/kg, i.p.	HFD-fed mice	Increased energy expenditure (Li et al., 2012)
	5% w/w for 4 weeks	C57BL/6N mice	Improved insulin sensitivity (Lin et al., 2012)
	400 mg/kg/day for 10 weeks; i.p	HFD + Low dose	Reduced insulin resistance (Khan and Jena, 2016a)
TSA	0.6 μg/kg/day for 12 weeks	HFD-fed mice	Reduced adiposity (Li et al., 2012)
	0.8 mg/kg, i.p.	HFD-fed mice	Induction of Fibroblast growth factor-21 (Li et al., 2012)
MS-275	10 mg/kg i.p.	C57BLKS/ J-Lepr^db/db^	Increased Energy expenditure; Increased insulin sensitivity (Galmozzi et al., 2013)
SAHA	25 mg/kg i.p. every other day for 23 days	C57BLKS/ J-Lepr^db/db^	Increased Energy expenditure; Increased insulin sensitivity (Galmozzi et al., 2013)
VPA	150–300 mg/kg/day for 3 weeks; orally	STZ (75 mg/kg, i.p.) in SD rats	Increased β-cell proliferation (Khan and Jena, 2016b)
	150–300 mg/kg/day for 10 weeks; orally	HFD + Low dose STZ	Reduced β cell damage; Reduced insulin resistance (Khan et al., 2016)
SAHA	25–50 mg/kg i.p.	Swiss albino mice fed with HFD for 8 weeks	Improved insulin resistance (Sharma and Taliyan, 2016b)
ITF 2357	1.25–2.5 mg/kg; orally	Female C57BL/6 mice	Reduced β cell toxicity; Decreases Serum Nitrite (Lewis et al., 2011)

### Histone Modification and Pancreatic β Cell Development and Function

Studies have shown that the modification of histones determines whether pluripotent pancreatic progenitor cells produce β cells. Haumaitre et al. studied the regulatory role of HDAC expression and activity in the development of rat pancreases and found that HDAC inhibitors can reduce the differentiation of pancreatic exocrine cells and increase the number of ductal cells and Ngn3-positive endocrine progenitor cells (Haumaitre et al., 2009). The dynamic changes in histone acetylation on the final different types of endocrine cells (that is, the number of α-, β-, δ-, ε-, and PP cells) have a decisive role. The different types of HDAC have different effects on the development of pancreatic cells. For example, class I HDAC members specifically inhibit the production of α- and PP cells while promoting the differentiation of β- and δ-cells (Haumaitre et al., 2008). The genetic deletion of different members of class II HDAC can lead to an increase in β cells and/or δ-cells, and their overexpression can cause the numbers of β- and δ-cells to be reduced (Lenoir et al., 2011). Therefore, histone modification enzymes have a highly specific role during the development and differentiation of different pancreatic cells. In addition, studies have shown that the HDAC inhibitor MC1568 can promote the expression of PDX4 and insulin (Dayeh and Ling, 2015). These results show that HDAC plays a key role in mediating pancreatic β cell differentiation and development.

A series of transcription factors, such as PDX1, require chromatin modification factors to effectively regulate gene transcription, which is essential for maintaining the normal function of β cells. If histone modification changes, it may cause a series of genes in β cells to exhibit high or low expression. This may further cause the occurrence of diabetes. Chakrabarti et al. found that β cells are highly methylated and acetylated at the H3K4 proximal promoter region of the insulin gene, and this modification is highly correlated with the recruitment of the histone methyltransferase Set7/9 and the histone acetyltransferase P300, which suggests that the expression of the insulin gene is regulated by histone modification (Chakrabarti et al., 2003). PDX1 can recruit the histone methyltransferase Set7/9, which in turn methylates H3K4 in the promoter region of the insulin gene, to promot the expression of the insulin gene (Maganti et al., 2015). Another study showed that Set7/9 is necessary for normal β cell function. Set7/9 can regulate insulin secretion-related genes (such as Ins1/2, Glut2, and MafA) with transcription factor PDX1 and RNA polymerase II (Deering et al., 2009). Related studies also show that under high glucose stimulation, p300 and PDX1 cooperate to promote insulin transcription of β cells; on the contrary, at low glucose levels, HDAC1 and HDAC2 bind to PDX1 to inhibit insulin transcription (Mosley and Ozcan, 2004; Wang et al., 2007). In addition, the Swi/Snf chromatin remodeling complex can be involved in the regulation of blood glucose by PDX1. Brg1-Swi/Snf can be used as a co-activator of PDX1-mediated gene expression in β cells, while Brm-Swi/Snf can be used as a co-suppression method. The antagonistic effects of Brg1-Swi/Snf and Brm-Swi/Snf affect the expression of target genes in β cells, which is important for maintaining glucose homeostasis. Chang et al. also found that PDX1 histone modification of the promoter region H3K4, such as deacetylation, demethylation and other histone modifications, can lead to downregulation of PDX1 in pancreatic β cells (Chang et al., 2016). Studies have also shown that MLL3 and MLL4 bind to the transcription factors MafA and MafB to regulate pancreatic β cell function (Scoville et al., 2015).

The article "Roles of Epigenetic Modifications in the Differentiation and Function of Pancreatic β-Cells" was retracted in 2022. Reasons: plagiarism; overlap with other authors' work.

The products of the Ink4a/Arf (Cdkn2a) locus, the cyclin-dependent kinase inhibitor p16INK4a and the tumor suppressor p19Arf showed increased expression with age and have been linked to reduction in the proliferative capacity of aged β cells (Krishnamurthy et al., 2006). The locus Cdkn2a has indeed been identified linked to T2DM by genome-wide association analysis (Diabetes Genetics Initiative of Broad Institute of et al., 2007). Interestingly, a recent study reported that Bmi-1 dependent modulation of the Ink4a/Arf expression levels is critical to regulate pancreatic β-cell proliferation during aging and regeneration (Dhawan et al., 2009). Loss of Bmi-1 resulted in reduced β-cell proliferation. Decreased Bmi- 1 binding to the Ink4a/Arf locus in aged islet led to reduced H2A ubiquitination. This epigenetic modification stimulated the recruitment of MLL1, a trithorax group (TrxG) protein, and increased H3K4me3 that augmented transcriptional activity from the Ink4a/Arf locus. During β-cell regeneration, increased Bmi-1 binding coincided with decreased H3K4me3, resulting in repression of the Ink4a/Arf locus and augmented β-cell proliferation.

The PcG protein Ezh2, functioning as a HMT in PolycombRepressive complex 2 (PRC2), was shown to regulate islet cell growth by influencing the proliferative potential of β cells (Chen et al., 2009). Conditional deletion of Ezh2 in β cells led to decreased H3K27me3 at the Ink4a/Arf locus. This induces a replication failure of β cells in neonatal mice, a reduced β- cell mass and mild diabetes. Ezh2, by regulating histone methylation and repression of the Ink4a/Arf locus in pancreatic islets, permit physiological β-cell expansion in neonatal mice, and adaptive β-cell regeneration after conditional chemical ablation of β cell in adults. This shows the importance of epigenetic mechanisms in the regulation of β-cell proliferation, and suggests that epigenetic manipulation of PcG proteins and their respective histone modification marks in β cells might be a useful tool for promoting β-cell proliferation. Altogether, these studies provide evidence that histone modifications, regulated by complexes containing TrxG and PcG proteins, are required for specific gene repression and permit physiological and adaptive β-cell expansion.

## The Role of Noncoding Rna in β Cell Differentiation and Function

### The Role of miRNAs in β Cell Differentiation and Function

MicroRNA is a type of endogenous noncoding small, single-stranded RNA of ~22 nucleotides in length. It is complementary to the site of the 3′ untranslated region of the target gene mRNA and binds through sequence-specific base pairing. The latest research shows that microRNA is closely related to pancreatic development, insulin secretion and insulin resistance, and may play an essential role in the pathogenesis of diabetes (Table 4) (Gilbert and Liu, 2012).

**Table 4:** miRNAs in the differentiation and function of pancreatic β cells.

**miRNAs**	**Targets**	**Functions**
miR-7	*GATA6, PDX6*	Regulate development and function of endocrine pancreas (Joglekar et al., 2011; Latreille et al., 2014)
	*Pfn2, Wipf2*	Regulate insulin secretion (Latreille et al., 2014)
	*Mknk2, Mknk1, eIF4E, S6k1*	Regulate the proliferation and differentiation of islet cells (Wang et al., 2013)
miR-375	*Mtpn, p38 MAPK, PI3K*	Promote the proliferation, differentiation and transdifferentiation of β cells (Ozcan, 2014)
	*CADM1, CAV1*	Regulate pancreatic development (Kloosterman et al., 2007)
	*PDK1*	Regulate the biosynthesis of insulin (Tang et al., 2007; El Ouaamari et al., 2008)
miR-9	*Onecut-2, SIRT1*	Inhibit insulin secretion (Plaisance et al., 2006)
miR-96	*NOC2*	Increase granuphilin/Slp4 and decrease Noc2
miR-15b, miR-16, miR-195, miR-106b	*Ngn3*	Regulate pancreatic development (Joglekar et al., 2007)
miR-21	*PTEN, PI3K, AKT*	Regulate pancreatic development (Ozcan, 2014)
miR-34a	*VAMP2, SNARE*	Decrease insulin production (Roggli et al., 2010)
miR-124a, let-7b	*PDX-1, Kir6.2, SUR1*, TGF-β / TGF-β-R pathway	Promote the differentiation of β cells (Ozcan, 2014)
miR-106b, miR-15a, miR-15b, miR-16, miR-195	*Ngn3*	Promote the formation of endocrine precursor cells (Joglekar et al., 2007)
miR-19b, miR-17-92/217	*NeuroD1*	Promotes the differentiation of pancreatic precursor cells into endocrine precursor cells (Taylor et al., 2013)
miR-18a, miR-145, miR-495	*Ptf1a*	Promotes the differentiation of pancreatic precursor cells into endocrine precursor cells (Krapp et al., 1998)
miR-29	*AMPK*	Inhibit pancreatic cell proliferation, promote apoptosis and autophagy (Pullen et al., 2011)
miR-145, miR-21	*Oct4, Sox2, Klf4*	Promote the differentiation of stem cells into human cells (Xu et al., 2009)
miR-290-295, miR-302	*Sox2*	Promote the differentiation of stem cells into human cells (Marson et al., 2008)
miR-182	*Rasa1, Grb2*	Maintain the stability of β cells (Melkman-Zehavi et al., 2011)
miR-23b	*Hes1*	Promote the differentiation of pancreatic endocrine cells (Ozcan, 2014)
miR-15a	*UCP2*	Regulate the biosynthesis of insulin (Sun et al., 2011)
	*Ngn3*	Regulate endocrine pancreas development and regeneration (Joglekar et al., 2007)
miR-30	*Vimentin, Snail1, Rfx6*	Regulate the proliferation and development of β cells (Liao et al., 2013)
	*Map4k4*	Regulate the biosynthesis of insulin (Zhao et al., 2012)
	*NeuroD*	Regulate insulin secretion (Kim et al., 2013)
miR-33a	*ABCA1*	Regulate insulin secretion (Roggli et al., 2010)
miR-130b	*SOX9, PDX6*	Maintain the number of pancreatic progenitor cells (Rosero et al., 2010)
miR-184	*Argonaute2*	Regulate compensatory amplification of β cells (Tattikota et al., 2014)
miR-200	*c-Maf, Fog2, Zeb, Sox17*	Regulate pancreatic differentiation (Liao et al., 2013)
miR-218, miR-495	*HNF6, Onecut2*	Regulate pancreatic development (Simion et al., 2010)
miR-342	*Foxa2, MafB, GATA4*	Regulate the proliferation and development of β cells (Kloosterman et al., 2007)
miR-382	*ISL1*	Regulate the differentiation and function of endocrine cells (Rosero et al., 2010)

*Pfn2, profilin 2; Wipf2, WAS/WASL interacting protein family member 2; eIF4E, eukaryotic translation initiation factor 4E; S6k1, Ribosomal protein S6 kinase 1; Mapkap1, MAPK associated protein 1; Mknk1, MAP kinase interacting serine/threonine kinase 1; Mknk2, MAP kinase; interacting serine/threonine kinase 2; SIRT1, silent information silent informationregulation 2 homolog-1; Onecut-2: one cut homeobox 2; UCP2, uncoupling protein 2; Ngn3, neurogenin 3; Ptf1a, pancreas associated transcription factor 1a; NeuroD1, neurogenic differentiation 1; SOX6, SRY-boxtranscription factor 6; SOX17, SRY-box transcription factor 17; MCT1, monocarboxylate transporter 1; Mcl-1, myeloid cell leukemia-1; Snail1, snail family transcriptional repressor 1; Map4k4, mitogen-activated protein kinase kinase kinase kinase 4; Abca1, ATP binding cassette subfamily A member 1; Zeb, zinc finger E-box binding homeobox; HNF6, hepatocyte nuclear factors 6; MafB, v-maf musculoaponeurotic fibrosarcomaoncogene homolog B; CADM1, cell adhesion molecule 1; PDK1, pyruvate dehydrogenase kinase 1; ISL1, islet1*.

miR-375 is the first miRNA found to be involved in glucose metabolism and is highly expressed in pancreatic islets. Poy et al. found that inhibiting endogenous miR-375 not only reduces insulin secretion but also affects the proliferation of pancreatic β cells (Joglekar et al., 2007). In mice lacking miR-375 (mi-375 knockout), the number of pancreatic islet alpha cells increased, and the number of pancreatic β cell clusters decreased, leading to increased blood glucose levels (Xu et al., 2009). PDX1 is one of the confirmed target genes of miR-375, and overexpression of miR-375 can downregulate PDX1 in the PI3-K pathway to reduce the expression of insulin genes and inhibit the proliferation of pancreatic β cells (Garikipati et al., 2017). Mir-375 also plays a regulatory role in the differentiation of islet cells. By analyzing the dynamic profile of the miRNA expression during the differentiation of iPSCs from hESCs, it was found that the expression of miR-375 increased at the early stage of iPSC differentiation and then decreased. In addition, miR-375 has a negative regulatory effect on the specific target genes HNFfl and Sox9 in the development of islet embryos to promote the differentiation and maturation of pancreatic β cells (Poy et al., 2004).

The article "Roles of Epigenetic Modifications in the Differentiation and Function of Pancreatic β-Cells" was retracted in 2022. Reasons: plagiarism; overlap with other authors' work.

Krek et al. found that miR-124a is highly expressed in MIN6 and has a synergistic effect with miR-375, which has been shown to jointly inhibit the myotrophin expression (Krek et al., 2005). FoxA2 is a well-defined miR-124a target gene that has important regulatory effects on pancreatic β cell differentiation and insulin secretion. Baroukh et al. found that miR-124a binds the FoxA2 mRNA 3′ UTR region, which can directly regulate the protein expression level of FoxA2 in pancreatic β cells (Baroukh et al., 2007). As the expression level of the FoxA2 gene decreases, the expression of downstream target genes increases, including PDX1, Kir6.2 and sulfonylurea receptor 1 (SUR1).

miR-7 is the most abundant miRNA expressed in the islets of humans and rats (Correa-Medina et al., 2009). It is highly expressed in the pancreatic islets of humans at 14–18 weeks of gestational age, a time at which the secretion of endocrine hormones by islets increases exponentially. Similar to miR-375, miR-7 is upregulated during the development and differentiation of human islets (Correa-Medina et al., 2009). Nieto et al. established a mouse model in which miR-7 was knocked out at embryonic E10.5. The synthesis of mouse insulin in the embryo was reduced and the number of pancreatic β cells was reduced (Nieto et al., 2012). MiR-7 is an important part of rapamycin complex 1 (mTORC1) and its down-stream effector S6K1 signaling, and the inhibition of mir-7a can activate mTOR signal to promote the proliferation of primary pancreatic β cells in adult mice (Wang et al., 2013).

miR-19 is an important member of the miR-17-92 gene cluster, which is highly enriched in pancreatic precursor cells, while its expression in pancreatic endocrine precursor cells shows a sharp downward trend in differentiated cells. This suggests that miR-19b is involved in the differentiation of pancreatic precursor cells into endocrine precursor cells. Further research shows that NeuroD is the target gene of miR-19b and that miR-19b can bind to the 3′-UTR sequence of NeuroD, which inhibits its expression and then downregulates the expression of the insulin gene (Yanaihara et al., 2006).

miR-9 can regulate Sirtl gene expression to regulate insulin secretion in pancreatic β cells (Ramachandran et al., 2011; Xu et al., 2013). In addition, miRNAs induced by inflammatory factors can mediate the death of pancreatic β cells, leading to insulin secretion defects. For example, the inflammatory factors TNFα and IL-1 in chronic inflammation can upregulate the expression of miR-21, miR-34a and miR-146, and these miRNAs in turn regulate the differentiation of pancreatic β cells and the insulin secretion. In addition, miR-30d, miR-15a, miR-24, miR-148a, and miR-182 also participate in the regulation of the expression of the insulin genes in pancreatic β cells (Melkman-Zehavi et al., 2011).

### The Role of lncRNAs in β Cell Differentiation and Function

LncRNA is a type of noncoding RNA with a transcription length greater than 200 nucleotides. Studies have found that lncRNAs are involved in the pathophysiological processes of diabetes, tumors, nervous system diseases and other diseases (Liu et al., 2016; Meng et al., 2017; Qi et al., 2017) LncRNA can combine with proteins to regulate downstream protein functions, or can be used as a structural component to form nucleic acid-protein complexes and bind to the promoter to regulate target gene transcription. Some lncRNAs serve as molecular sponges to bind miRNAs, reducing miRNA bioavailability and regulate the expression of target genes (Table 5) (Guay et al., 2012; Xin et al., 2017).

The article "Roles of Epigenetic Modifications in the Differentiation and Function of Pancreatic β-Cells" was retracted in 2022. Reasons: plagiarism; overlap with other authors' work.

**Table 5:** lncRNAs and circRNAs in the differentiation and function of pancreatic β cells.

**LncRNAs or circRNAs**	**Location**	**Targets**	**Functions**
KCNQ1	11p15.5	CDKN1C	Regulate the proliferation and development of β cells (Avrahami et al., 2014)
H19	11p15.5	IGF2	Regulate insulin secretion (Hark et al., 2000; Schoenherr et al., 2003)
MEG3	14q32	DLKl, RTL1	Regulate the biosynthesis of insulin (Kameswaran et al., 2014)
PLUT	13q12.2	PDX1	Regulate the development of β cells and insulin secretion (Yin et al., 2015)
TUG1	22q12.2	/	Regulate the biosynthesis and secretion of insulin (Yin et al., 2015)
H1-LNC25/ LINC01370	20q12	Glis	Regulate the development of β cells (Ravassard et al., 2011)
CDR1as	Xq27.1	miR-7	Promote development and function of endocrine pancreas; promote insulin secretion (Hansen et al., 2013)
circHIPK3	11p13	miR-338-3p, miR-124-3p	Promote the proliferation and development of β cells; promote insulin secretion (Stoll et al., 2018)

#### KCNQ1 Gene

The KCNQ1 gene is one of the members of the voltage-dependent potassium channel family (Splawski et al., 1998). The gene is located at 11p15.5, nearing the imprinting site H19-IGF2 (Hussain et al., 2005). This imprinting region includes some conserved maternally expressed protein-coding genes, such as Cyclin-dependent kinase inhibitor 1C (CDKN1C) and the paternal lncRNA KCNQ1 overlapping transcript 1 (KCNQ1OT1) (Monk et al., 2006). Loss of this imprinting site can lead to inhibition of CDKN1C, causing β cells to re-enter the cell cycle and resulting in increased insulin levels and decreased blood glucose levels (Avrahami et al., 2014).

Unoki et al. applied the genome-wide associate study (GWAS) method to conduct a comprehensive screening of 207,097 single nucleotide polymorphisms (SNPs) and analyzed the genetic polymorphisms of the T2DM group and the healthy control group (Unoki et al., 2008). The risk of T2DM is significantly related to 6 SNPs (rs2237897, rs2237896, rs2299620, rs2237895, rs227892, and rs163171), which can triple the risk of T2DM (Travers et al., 2013). The risk allele of homozygous rs2237895 in fetal samples increased slightly in the KvDMR region but was not observed in adults because KCNQ1 and KCNQ1OT1 are expressed in only the fetus (Travers et al., 2013). These results indicate that the risk allele may be in the islets. In the early stages of development, this study proposed a model in which the risk allele of the rs2237895 SNP led to an increase in KvDMR methylation, which resulted in a decrease in KCNQ1OT1 expression. However, KCNQ1OT1 expression did not differ significantly between the T2DM and control groups. In contrast, the transcription level of KCNQ1OT1 was significantly increased in the islet of the pancreas in T2DM, which was associated with an overall decrease in CpG methylation of the KCNQ1 gene (Moran et al., 2012). Therefore, the pathological interpretation of the variants in this region has always been a contradiction and challenge. However, the regulation of this site and lncRNA KCNQ1OT1 is still closely related to the pathogenesis of β cell biology and T2DM, and the mechanism needs further study.

The article "Roles of Epigenetic Modifications in the Differentiation and Function of Pancreatic β-Cells" was retracted in 2022. Reasons: plagiarism; overlap with other authors' work.

#### H19/IGF2 Gene Locus

The H19/IGF2 gene locus is located on chromosome 11p15.5 adjacent to KCNQ1, and includes the IGF2 gene expressed by the male parent and the H19 lncRNA expressed by the female parent (Brannan et al., 1990). The former is essential for early embryonic development, while the latter can inhibit tumors (Hao et al., 1993). The imprinting control region (ICR) is located between these two genes. On the maternal chromosome, the ICR is unmethylated and binds to the transcription factor CCCTC (CTCF). This interaction has an insulator function to block the downstream enhancer from binding to the IGF2 gene promoter so that the downstream enhancer instead acts on the H19 promoter and promotes H19 expression. Because the ICR is methylated on the chromosome, it cannot bind to the CTCF transcription factor and cannot act as an insulator. Therefore, the downstream enhancer cannot bind to the H19 gene promoter, but instead binds only to the IGF2 gene promoter. Thus, the downstream enhancer inhibits the expression of the H19 gene and promotes the expression of IGF2 (Hark et al., 2000; Schoenherr et al., 2003).

Loss of ICR methylation at the H19/IGF2 locus inhibits IGF2 expression, which can cause syndromes of short stature and low birth weight in rodent models and humans; one example is Silver-Russell syndrome, which is a characteristic developmental disorder characterized by retardation of intrauterine and postpartum growth (DeChiara et al., 1990). To ensure the development of important organs, metabolic processes in fat, skeletal muscle and other peripheral tissues can undergo permanent changes and lead to insulin resistance. This observation is called the “thrifty phenotype hypothesis.” However, Ding et al. found that impaired glucose tolerance in the progeny of mice with GDM is accompanied by H19 ICR hypermethylation in islets (Ding et al., 2012). This contradictory finding may be caused by exposure of the developing fetus to different nutritional states or by different exposure times. The above studies show that the H19/IGF2 gene locus can respond to the intrauterine environment and can be used to predict future metabolic complications.

The article "Roles of Epigenetic Modifications in the Differentiation and Function of Pancreatic β-Cells" was retracted in 2022. Reasons: plagiarism; overlap with other authors' work.

Hypermethylation of the H19/IGF2 ICR can be found in some patients with Beckwith-Wiedemann syndrome (BWS) and focal congenital hyperinsulinaemia (FoCHI); the latter is a glucose metabolism disease characterized by abnormal insulin secretion by pancreatic β cells and hypoglycaemia (Ohlsson et al., 1993). ICR hypermethylation can lead to a decrease in H19 expression and an increase in IGF2 expression. Devedjian and Fournet et al. found that although IGF2 was overexpressed in mouse FoCHI model, expression in the human FoCHI model was different; however, H19 transcription was consistently downregulated, indicating that H19 has a very important regulatory role in inhibiting the proliferation of pancreatic β cells (Devedjian et al., 2000; Fournet et al., 2001). This type of ICR hypermethylation with decreased expression of H19 has also been reported in nephroblastoma. As mentioned previously, the lncRNA H19 regulates β cell function and cell proliferation, and its level can be adjusted independently or indirectly by adjusting the level of IGF2.

#### DLK1/MEG3 Gene Cluster

DLK1-MEG3 gene cluster is located on chromosome 14q32 in humans (chromosome 12 in mice) and includes paternally expressed protein-coding genes, such as DLK1, RTL1, and DIO3, and maternally expressed non-coding RNAs, such as MEG3, miRNAs, and snoRNAs. DLK1 is expressed in many embryonic tissues and is a negative regulator of adipocyte differentiation. It is highly expressed in human and mouse β cells (Appelbe et al., 2013). This cluster is strictly regulated by the ICR, which consists of two paternal differentially methylated regions (DMR). One region called IG-DMR, which is the primary ICR, is located at 13 kb upstream of the MEG3 transcription start site. The other region overlaps with the MEG3 multi-cis-trans acting transcription site promoter, called the MEG3-DMR. Deletion of this imprinted area can lead to maternal or paternal diploidy of chromosome 14 (uniparental disomy, UPD), thereby causing various severe developmental disorders.

A recent study revealed that the non-coding RNA of the DLK1/MEG3 imprinting site is downregulated in the islets of T2DM patients, but the specific mechanism is unclear (Kameswaran et al., 2014). Increased methylation of the MEG3/DMR and decreased expression of MEG3 can also be observed in some cancers, such as pituitary cancer, renal cell carcinoma, and multiple myeloma. *In vitro* experiments have further revealed that MEG3 can exert tumor suppressive effects by activating the p53 gene; these functions are partially dependent on the secondary structure of the MEG3 RNA. In addition, the decrease in MEG3 expression in T2DM may be closely related to increased methylation of the MEG3/DMR.

The article "Roles of Epigenetic Modifications in the Differentiation and Function of Pancreatic β-Cells" was retracted in 2022. Reasons: plagiarism; overlap with other authors' work.

#### LncRNA PLUT

The lncRNA Pdx1-associated lncRNA upregulator of transcription (PLUT) is abundantly expressed in the nucleus of islet β cells, and its enhancer region can bind to the promoter of the key pancreatic β cell transcription factor PDX1 to participate in regulating pancreatic islet β cell transcription and differentiation processes (Yin et al., 2015). PDX1 can induce endoderm cells to develop and mature into pancreatic cells and can further induce their differentiation into insulin-secreting cells. On the other hand, PDX1 is also involved in mediating insulin transcription factors and glucose transport, which is important in the development of the pancreas and in the regulation of insulin secretion. Therefore, loss of the lncRNA PLUT, leads to downregulation of PDX1 expression, will lead to abnormal development of the pancreas.

#### LncRNA TUG1

Pancreatic β cells are the main insulin-producing cells, but they are also regulated by insulin and dysfunction of these cells is a key process in the development of T2DM. Studies have shown that lncRNAs are involved in regulating the secretory function of pancreatic β cells. The lncRNA TUG1 is expressed in β cells. Yin et al. silenced the TUG1 gene in adult non-obese diabetic (NOD) mice via siRNA transfection and found that islet β cell synthesis and insulin secretion were significantly reduced, while islet β cell apoptosis was increased (Yin et al., 2015). This pattern suggests that TUG1 may be involved in maintaining islet β cell function and may play an important role in glucose metabolism homeostasis. High-glucose conditions further inhibit the expression of the TUG1 gene in pancreatic β cells, causing a vicious cycle and triggering diabetes.

#### lncRNA H1/LNC25

LncRNA H1/LNC25 is a multifunctional exon transcript cluster that is highly expressed in pancreatic β cells and participates in the regulation of insulin secretion. Studies have shown that the expression of lncRNA H1/LNC25 in pancreatic β cells of diabetic patients is significantly reduced (Ravassard et al., 2011). Moran et al. found that the expression of Glis family zinc finger 3 (Glis3) mRNA was significantly reduced upon the inhibition of lncRNA H1/LNC25 expression in human pancreatic β cells (Moran et al., 2012). Glis3 is a member of the Glis-like zinc finger family and encodes an insulin transcription factor. Loss of Glis3 expression causes the insulin secretion of pancreatic β cells to decrease (Nogueira et al., 2013). Therefore, it can be speculated that the lncRNA H1/LNC25 affects glucose metabolism by affecting the expression of Glis3, which in turn leads to the occurrence of diabetes.

The article "Roles of Epigenetic Modifications in the Differentiation and Function of Pancreatic β-Cells" was retracted in 2022. Reasons: plagiarism; overlap with other authors' work.

In summary, lncRNAs, which are key factors regulating the homeostasis of glucose metabolism homeostasis, play important roles in the developmental regulation and function of islet β cells development and biological function. A single lncRNA can act through multiple pathways, and multiple lncRNAs can also act together within the same pathway. Although the current understanding of lncRNAs is insufficient, detection detecting the expression of specific lncRNAs expression in tissues or body fluids may be a new means of approach to predicting the risk of diabetes. The discovery of additional lncRNAs will provide us with more comprehensive ways to improve models for research on glucose metabolism homeostasis research models.

### Roles of Circular RNAs (circRNAs) in β Cell Differentiation and Function

CircRNAs are closed, circular, non-coding RNAs that do not have 5' caps or 3′ poly(A) tails, are not easily degraded by exonucleases, and have the characteristics of structural stability, tissue specificity, and evolutionary conservation (Stoll et al., 2018). CircRNAs can be divided into three categories according to their sources: exonic circRNAs (e-circRNAs), intronic circRNAs (ciRNAs), and exonic/intronic circRNAs (EIciRNAs) (Stoll et al., 2018; Li R. et al., 2019). With the rapid development of high-throughput sequencing and other biotechnologies, numerous circRNAs have been found in various organisms, such as nematodes, fruit flies, mice, macaques, and humans. Further studies have revealed that circRNAs play important roles in the occurrence and development of cancer, nervous system diseases, cardiovascular diseases, and metabolic diseases (Wang et al., 2019; Xiao, 2020).

Hansen et al. believed that CDR1as could negatively regulate miR-7 through sponging miR-7, suppress the inhibitory effect of miR-7 on the mTOR signaling pathway, and stimulate pancreatic β cell proliferation and insulin secretion (Hansen et al., 2013). The study showed that circHIPK3 was downregulated in the islets of diabetic model mice which inhibited β cell proliferation and insulin secretion. The mechanism may involve the competitive interaction of circHIPK3 with miR-338-3p and miR-124-3p to regulate the key genes in the development, proliferation and function of pancreatic β cells, such as glucose transporter 2 (Glut2) and protein kinase B1 (PKB1) (Stoll et al., 2018). Zhao et al. found 489 circRNAs differently expressed in the peripheral blood of T2DM patients. They further verified that circRNA-0054633 (hsa_circ_0054633) could be used as a diagnostic marker for T2DM (Zhao et al., 2017). Hsa_circ_0054633 is not only involved in biological processes such as cell cycle and mitotic arrest but is also closely related to the pathogenesis of diabetes mellitus (Werfel et al., 2016; Zhao et al., 2017). By collecting peripheral blood of patients with T2DM, coronary heart disease, T2DM complicated with coronary heart disease and health group, the results of circRNA microarray showed that HAS-cirC-11783-2 was closely related to T2DM and coronary artery disease (Salzman et al., 2013).

The article "Roles of Epigenetic Modifications in the Differentiation and Function of Pancreatic β-Cells" was retracted in 2022. Reasons: plagiarism; overlap with other authors' work.

Although accumulating studies have indicated that circRNAs play key regulatory roles in the occurrence and development of diabetes, the more specific biological functions and molecular mechanisms need to be further revealed.

## Conclusion

Epigenetic regulation of pancreatic islets is of major interest to understand how endocrine cells differentiate, proliferate, establish, and maintain their mature identity and function. The development process of β cells from multipotent progenitors can be successfully recapitulated only partially *in vitro* to generate pancreatic progenitors and functional β cells in cell replacement therapy for treating diabetes. Thus, the epigenomic study of pancreatic islets cells has become a necessity to overcome the barriers that restrict lineage plasticity and is an exciting prospect for the future development of successful β-cell differentiation strategies (Balaji et al., 2018; Lv and Huang, 2019; Scarpa, 2019; Gong and Jiang, 2020). Dissecting the epigenetic components of islet cell-specific transcriptional networks would contribute to induce and maintain appropriate endocrine lineage commitment from embryonic stem cells or induced pluripotent cells. Knowledge and manipulation of the PcG-repression and derepression programs of pancreatic progenitors and β cells would provide benchmarks to direct β cell differentiation protocols. Epigenetic manipulations demonstrated the importance of DNA methylation and histone modifications in maintaining β-cell identity and driving islet cell differentiation. They have underscored the potential of using reprogramming methods to change identity or regain plasticity of adult endocrine cells and generate novel sources of islet cells. It is also expected that the better understanding of the epigenetic mechanisms leading to enhanced β-cell mass, or to β-cell proliferation and function defects during diabetes, allows identification of novel therapeutic targets. A detailed understanding of the specialized functions of epigenetic regulators in healthy and diabetic islets, together with the generation of specific compounds targeting these components, may accelerate development of strategies for islet replacement or regeneration therapies for prevention and treatment of diabetes.

The article "Roles of Epigenetic Modifications in the Differentiation and Function of Pancreatic β-Cells" was retracted in 2022. Reasons: plagiarism; overlap with other authors' work.

## Author Contributions

FX and JL conceived and designed the study. FX and LN performed the data collection and analysis. FX and LC interpreted the data and wrote the manuscript. All authors read and approved the final manuscript.

## Conflict of Interest

The authors declare that the research was conducted in the absence of any commercial or financial relationships that could be construed as a potential conflict of interest.
